The article "MicroRNA‐181b negatively regulates the proliferation of human epidermal keratinocytes in psoriasis through targeting TLR4" was retracted in 2021. Reasons: errors in the data; errors in the analysis; errors in the results or conclusions.

# MicroRNA‐181b negatively regulates the proliferation of human epidermal keratinocytes in psoriasis through targeting TLR4

**DOI:** 10.1111/jcmm.12963

**Published:** 2016-09-19

**Authors:** Cheng Feng, Ming Bai, Nan‐Ze Yu, Xiao‐Jun Wang, Zeng Liu

**Affiliations:** ^1^ Aesthetic Plastic Department of Peking Union Medical Collage HospitalBeijingChina

**Keywords:** microRNA‐181b, keratinocytes, psoriatic lesions, psoriasis, *TLR4*, immunohistochemistry, qRT‐PCR, Western blotting

## Abstract

Our study aims to explore the role of microRNA‐181b (miR‐181b) and TLR in the regulation of cell proliferation of human epidermal keratinocytes (HEKs) in psoriasis. Twenty‐eight patients diagnosed with psoriasis vulgaris were selected as a case group with their lesional and non‐lesional skin tissues collected. A control group consisted of 20 patients who underwent plastic surgery with their healthy skin tissues collected. Real‐time quantitative fluorescence polymerase chain reaction (RT‐qPCR), *in situ* hybridization and immunohistochemistry were used to detect the expressions of miR‐181b and TLR4 in HEKs of healthy skin, psoriatic lesional skin and non‐lesional skin respectively. The 3′ untranslated region (3′UTR) of TLR4 combined with miR‐181b was verified by a dual‐luciferase reporter assay. Western blotting and bromodeoxyuridine were applied for corresponding detection of TLR4 expression and cell mitosis. The expression of miR‐181b in HEKs of psoriatic lesional skin was less than healthy skin and psoriatic non‐lesional skin. In psoriatic lesional and non‐lesional skin, TLR4‐positive cell rates and the number of positive cells per square millimetre were higher than healthy skin. The dual‐luciferase reporter assay verified that miR‐181b targets TLR4. HEKs transfected with miR‐181b mimics had decreased expression of TLR4, along with the decrease of mitotic indexes and Brdu labelling indexes. However, HEKs transfected with miR‐181b inhibitors showed increased TLR4 expression, mitotic indexes and Brdu labelling indexes. HEKs transfected with both miR‐181b inhibitors and siTLR4 had decreased mitotic indexes and Brdu labelling indexes. These results indicate that miR‐181b can negatively regulate the proliferation of HEKs in psoriasis by targeting TLR4.

## Introduction

Psoriasis is a chronic inflammatory disease of the skin 1. According to the worldwide statistic, the prevalence rates of psoriasis, ranging from 0.6 to 4.8%, tend to be a bimodal distribution of onset with the major peak and a later smaller peak at the age of 20–30 and 50–60 respectively 2. The subgroup for this disease mainly includes psoriasis vulgaris (also called plaque psoriasis), pustular psoriasis, psoriatic arthritis and erythrodermic psoriasis clinically 3, 4, characterized by excessive growth of the epidermal layer of the skin, chronic inflammation in the dermis and parakeratosis 5. Currently, the aetiology of psoriasis is not fully understood, but genetics, cell apoptosis and proliferation, immunity, inflammation and neurotransmitters are reported to be involved 6, 7, 8. Although typical medications of psoriasis involve retinoid acids 9, methotrexate 10, cyclosporine 11, compound glycyrrhizin 12, few of them have targeting effects because of the complexity of psoriasis. Currently, the discovery of new immunological factors and a more comprehensive understanding of psoriasis promote the application of immunological pathways. In this regard, new biological drugs against specific immunological elements that cause psoriasis may be available 13. As a well‐established treatment modality, the combination use of photodynamic therapy (PDT) with immunomodulation has been shown to be effective and safe for many skin disorders, including psoriasis 14. Moreover, based on further clinical and pathological studies, some novel drugs targeting microRNA (miR) have been arisen for improvement of drug efficacy 15, 16, 17.

The miRs, widely found in eukaryotes, are a group of small (~19–24 nucleotides) and non‐coding RNAs that interfere with protein components and protein factors relevant to chromosomal rearrangements, and that inhibit translation of the promoter region, by specifically interacting with the corresponding target genes, which results in gene expression silence and plays critical roles in gene regulation 18. In recent years, with the comprehensive genetic analysis on miR, increasing numbers of specific miR have been discovered to be related with the pathology of psoriasis 19, including miR‐21 20, miR‐146a 21, miR‐424 22 and miR‐99a 23. Other previous studies have also shown that miR‐203, miR‐125b, miR‐99a and miR‐197 were relevant to the pathogenesis of psoriasis by regulating target genes 24, 25, 26, 27. The miR‐181 family includes miR‐181a, miR‐181b, miR‐181c and miR‐181d, commonly existing in human cells 28. The miR‐181 members are involved in growth and development of immune cells like T and B cells, participating in pathological processes of various diseases, such as immune responses, immune tolerance and inflammatory responses 29, 30. But the role of miR181‐b in mechanisms underlying psoriasis has not yet been studied so far. On the other hand, Toll‐like receptors (TLRs) of epidermal cells are transmembrane proteins, with the extracellular portions or the intracellular portions conjugated to corresponding ligands, capable of initiating innate immune responses and influencing subsequent adaptive immune responses 31, 32. Evidence supported that TLR4 in immune response has been revealed in the pathogenesis of psoriasis 33, and increased gene expression of TLR4 on peripheral blood mononuclear cells in patients with psoriasis was revealed 34. In addition, although the negative correlation of TLR4 with miR181‐b has been revealed in a previous study in acute myeloid leukaemia 35, whether such a correlation was still existed in on psoriasis pathogenesis remains unexplored. Therefore, this study aims to investigate the roles of miR‐181b and TLR in the regulation of cell proliferation of human epidermal keratinocytes (HEKs) in psoriasis, so as to search for influential factors and new treatments for psoriasis.

## Material and methods

### Participants

From August 2013 to June 2015, 28 patients diagnosed with psoriasis vulgaris in Aesthetic Plastic Department of Peking Union Medical Collage Hospital were recruited as a case group. The inclusion criteria were: (i) Patients were withdrawn from systemic antipsoriatic drugs (including oral corticosteroids, immunosuppressants, antimalarials, receptor inhibitors, herbs) for at least a month, (ii) No topical treatment was employed within a month, (iii) Included patients had no immune and neoplastic diseases. There were 18 male and 10 female patients in the case group, ageing from 15 to 60 years old with the average age of 36.8 years old. Lesional skin and non‐lesional skin (0.5 cm away from the lesional skin area) were taken from the trunk or limbs of each patient. The control group was consisted of 20 cases of healthy skin tissues taken from patients who underwent plastic surgery in Aesthetic Plastic Department of Peking Union Medical Collage Hospital, including 11 men and 9 women who aged from 15 to 48 with the average age of 32.4 years. There was no significant difference in the age and sex between the two groups (both *P* > 0.05). Tissues (4 mm) were cut for biopsy and these isolated samples were immediately preserved in liquid nitrogen for subsequent analysis. The study was approved by the Institutional Review Boards of Aesthetic Plastic Department of Peking Union Medical Collage Hospital and the written informed consent was obtained from each eligible participant.

### *In situ* hybridization (ISH)

ISH is the application of molecular hybridization in gene localization. The cut and prepared frozen sections were hydrated in PBS solution for 10 min., then immersed in H_2_O_2_ for an extra 15–25 min. and rinsed by PBS for 3 times. Each section was then treated with a drop of pepsin solution and washed by PBS for 3 times. After the addition of pre‐hybridization solution, sections were incubated in a humid box at 37°C for 2 h, followed by the rinsing process using 2 × SSC at 37°C for 5 min. The probe mixture was denatured at 65°C for 5 min. and diluted into 40 nM by the pre‐hybridization solution, before being added to sections which were then hybridized at 52°C overnight and washed by 0.2 × SSC for 3 times next day. Then, sections were blocked using the blocking buffer at room temperature for 30 min. One drop of peroxidase (POD) chromogenic agent was added to each section and sections were kept at 37°C for 40 min. before being rinsed by PBS for 3 times. Colorization was realized using the 3, 3′‐diaminobenzidine (DAB) chromogenic agent. The locked nucleic acid (LNA) probes specifically recognizing miR‐181b in the experimental group and the probes of the negative group were purchased from a Danish company, EXIQON. The qRT‐PCR assay was used to evaluate the changes of miR‐181b expression in HEKs, keratinocytes.

### Immunohistochemistry

The frozen sections were incubated in 3% H_2_O_2_ at room temperature for 10 min. to block endogenous peroxidase activity and then immersed in the citrate buffer (pH 6.0) for following antigen retrieval under high pressures. After the PBS wash step, normal non‐immune animal serum was added and removed later, followed by the addition of TLR4 antibodies (ab47093, Abcam, USA) (diluted in the proportion of 1:150). Sections were incubated at 4°C overnight and rinsed by PBS next day. Each section was treated with biotinylated secondary antibodies (Abcam Inc., Cambridge, MA, USA) before 15‐min. incubation at room temperature. They were then washed by PBS and treated with streptavidin‐peroxidase solution. Upon the PBS rinse step, DAB was applied for colour developing. Sections were counterstained with haematoxylin, dehydrated an ethanol series, cleared by xylene and sealed with neutral gum. Results were observed under microscopes. In this experiment, rabbit non‐specific IgG was employed as the negative control, replacing the primary antibody for interpretation of the results. Positive expression of TLR4 was located in cytoplasm, shown as brown granules. For each slide, 10 microscopic fields under high‐power magnification were randomly chosen, and 100 cells in every field were counted and scored according to intensity of stain 36. The extensional standards were: (i) intensity of stain: colourless, scored 0; pallide‐flavens, scored 1; yellow, scored 2; brown, scored 3; (ii) percentages of positive stained cells: <5%, scored 0; 5–25%, scored 1; 26–50%, scored 2; 51–75%, scored 3; >75%, scored 4. Multiply (i) and (ii) and the staining scores were stratified as a negative result (0–3 score) and a positive result (≥4 score). The numbers of positive stained cells per square millimetre were counted in five randomly picked microscopic fields (10 × 40), with the mean calculated.

### Cell isolation and culture

Tissue specimens were washed by PBS for removal of blood stains, disinfected with iodophor and extensively washed with PBS. The specimens were then minced into 0.5 cm × 0.5 cm and digested with 0.25% trypsin overnight. After digestion for 24 h, the specimens were manually separated the epidermis from the dermis 37 and then the epidermis was taken and digested into single cells with 0.25% trypsin. Cells were grown and maintained in Epilife medium at 37°C in a humidified atmosphere of 5% CO_2_. The cell culture medium was changed every other day until the moment when cells were grown to 70% confluence and passaging started. Upon 2–3 passaging, purified HEKs were obtained and the third or fourth passage cells after verification were selected for subsequent studies.

### Dual‐luciferase reporter assay

The recombinant plasmids of wild‐type and TLR4 mutant (pMIR‐Report/wt‐TLR4 and pMIR‐Report/mut‐TLR4) were constructed and extracted by the EndoFree Plasmid Maxi Kit. Corresponding expression vectors and interference vectors were constructed by Shanghai GenePharma Co., Ltd. The experimental group included pMIR‐Report/wt‐TLR43′UTR and miR‐181b analogues or the negative control of miR‐181b sequence. The control group included pMIR‐Report/mut‐TLR4 3′UTR and miR‐181b analogues or the negative control of miR‐181b sequence. Liposome Lipofectamine2000 was applied to co‐transfect HEKs. According to the specification of dual‐luciferase reporter kit (Dual‐Luciferase Reporter Assay System Promega, Madison, WI, USA), the procedures described were: (i) Medium in the 96‐well plate was removed and the plate was washed by PBS for 3 times. (ii) Each well of the plate was treated with 20 μL 1 × passive lysis buffer (PLB) and placed in a constant temperature air bath for 15 min. before detection; (iii) The programme was set (2 sec. as an interval, reading at 10 sec.). Each well of the plate was treated with 50 μL luciferase assay substrate and 50 μL Stop&Glo substrate in sequence, with both sets of data collected automatically and analysed.

### Design and synthesis of TLR4‐siRNA

The siRNA software from Invitrogen were applied for TLR4‐siRNA design based on TLR4 mRNA sequence (NM 001082732) (as shown in Table 1). The target sequence for siRNA sequence includes 21 basic groups with G/C of approximately 50%. Those sequences applied were homology compared using BLAST analyses without any repetitive sequences with other genes. The TLR4‐siRNA was synthesized and modified by Guangzhou RiboBio (RiboBio, China).

**Table 1:** The sequences for TLR4 silencing and miR‐181b qRT‐PCR assay

Gene	Sequences
TLR4	Sense: 5′GATCCGACCATCATTAGCGTGTCATTCAAGAGATGACACGCTAATGATGGTCTTTTTTGGAAA 3′
	Anti‐sense: 5′AGCTTTTCCAAAAAAGACCATCATTAGCGTGTCATCTCTTGAATGACACGCTAATGATGGTCG 3′
microRNA‐181b	Sense: 5′‐ACACTCCAGCTGGGAACATTCATTGCTGTCGG‐3′
	Anti‐sense: 5′‐TGGTGTCGTGGAGTCG‐3′

qRT‐PCR, real‐time quantitative fluorescence polymerase chain reaction.

### Cell transfection

Cells were classified into (a) miR‐181b inhibitor group; (b) LZRs group; (c) blank group; (d) miR‐181b inhibitor + siTLR4 group; (e) miR‐181b mimic group. Keratinocytes isolated from healthy skin were inoculated in a 24‐well plate with a density of 2 × 10^5^ cells per well, and cultured at 37°C with 5% CO_2_ for 24 h. Liposome‐mediated DNA, miR‐181b inhibitor (German QIAGEN) and siTLR4 were diluted with 10 μL of serum‐free DMEM medium respectively and then 100 μL of each mixture was added into each well. Cells were then cultured under the conditions of 37°C, 5% CO_2_ and saturated humidity for 6 h, transferred to the fresh DMEM medium containing 10% FBS for 48 h and preserved for the subsequent studies.

### Real‐time quantitative fluorescence polymerase chain reaction (qRT‐PCR)

The amplification and melting curve analysis of qRT‐PCR reactions were performed with ABI 7500PCR (Applied Biosystems, Foster City, CA, USA). The RT primer sequences of miR‐181b were shown in Table 1. The volume of the reverse transcription reaction system was 5 μL (Total RNA 1.0 μL, 5 × RT buffer 2.0 μL,primer mix (10 μM) miR‐181b primer 0.5 μL, U6 primer 0.5 μL, RT enzyme mix 0.5 μL,nuclease‐free water 0.5 μL) and reaction conditions were 42°C for 60 min., 70°C for 15 min. and holding at 4°C. Obtained 1 μL of cDNA was added into the 25 μL reaction system of qRT‐PCR (cDNA 1.0 μL, sense primer (10 μM) 0.5 μL, anti‐sense primer (10 μM) 0.5 μL, SYBR Green real‐time PCR master mix 12.5 μL, nuclease‐free water 10.5 μL) and reaction conditions were 50°C for 2 min. for initial denaturation, 95°C for 2 min., 95°C for 15 sec. and 60°C for 30 sec., followed by 40 cycles of amplification. The melting curve analysis was conducted under the conditions of 95°C for 15 sec., 60°C for 1 min., 85°C for 15 sec. and 60°C for 15 sec. Glyceraldehyde 3‐phosphate dehydrogenase (GAPDH) was used as the reference and each sample was measured in triplicate. Results of qRT‐PCR were processed based on the 2^−ΔΔCt^ method. The values of threshold were manually set at the lowest points of the parallel rises of corresponding exponential amplification curves with the threshold cycle (Ct) values calculated. The relative gene expressions between the experimental group and the control group were determined by calculating 2^−ΔΔCt^ following the equations (ΔΔCt_target gene_ = ΔCt_target gene_−ΔCt_reference gene_, ΔCt_target gene_ = Ct_target gene_−Ct_reference gene_) 38.

### Western blotting

Western blotting was performed as described in the previous experiment. TLR4 and GAPDH antibodies were purchased from Santa Cruz Biotechnology and Abcam respectively. The prepared protein samples were separated by SDS‐PAGE electrophoresis and the gel was removed from the mould. Several pieces of filter paper, a nitrocellulose membrane, the gel and some filter paper were placed sequentially from the bottom to the top and any air bubbles trapped between layers were rolled out before this stack underwent the procedure of transfer in the electrophoresis apparatus for 1.5 h. When the transfer was complete, the nitrocellulose membrane was washed by phosphate‐buffered saline with Tween 20 (PBST) and immersed in 5% non‐fat dried milk on a shaker at room temperature for 2 h. It was then treated with rabbit anti‐human TLR monoclonal antibodies (1:1000), incubated at 4°C overnight and rinsed for 4 × 10 min. with PBST next day, followed by being incubated in horseradish peroxidase conjugated goat anti‐rabbit secondary antibodies (1:4000) on a shaker at the temperature for 2 h. After the PBST rinse step, it was stained *via* chemiluminescence detection using ECL.

### Bromodeoxyuridine (BrdU) staining

Cells were incubated with 10 μM BrdU for 1 h and for an extra hour after the transfer to fresh medium, and then fixed with paraformaldehyde. PBS containing 0.01% BSA and 0.01% Tween‐20 was used at the blocking step for 1 h and BrdU antibodies (1:10, Developmental StudiesHybridoma Bank) were added for 30‐min. incubation, with excess antibodies removed by PBS. After the 1 h incubation with HPR‐modified secondary antibodies, cells were washed with PBS followed by colour development.

### Statistical analysis

SPSS 21.0 software was used for statistical analysis. Measure data were expressed by mean ± standard deviation ($\overset{¯}{x}$ ± SD) and analysed by the normality test. The two groups were compared using the *t*‐test and the multiple groups were compared using one‐way analysis of variance (anova) (the homogeneity test of variances was done before this analysis) with means among multiple groups compared in pairs using the least significant difference (LSD) *t*‐test. Count data were compared among groups using the *I* ^2^ test. *P* < 0.05 showed significant difference.

## Results

### Expression of miR‐181b in psoriasis

The expressions of miR‐181b in health skin (n = 20), psoriatic lesional skin (n = 28) and non‐lesional skin (n = 28) were detected by ISH using miR‐181b specific probes. As shown in Figure 1A, miR‐181b, confined in HEKs of the suprabasal layer of the epidermis in healthy skin tissues, was highly expressed, while its expression decreased in HEKs of both the basal and suprabasal layers in psoriatic non‐lesional skin. In psoriatic lesional skin tissues, the expression of miR‐181b, mainly in HEKs of the basal layer, experienced a further decrease. The qRT‐PCR results showed that the expression of miR‐181b in HEKs of psoriatic lesional skin was less than that of healthy skin and psoriatic non‐lesional skin (both *P* < 0.05) (Fig. 1B).

**Figure 1:** The expressions of miR‐181b in psoriatic lesional skin, non‐lesional skin and healthy skin.**(A)** the expressions of miR‐181b in psoriatic lesional skin, non‐lesional skin and healthy skin were detected by *in situ* hybridization. **(B)** the expressions of miR‐181b in psoriatic lesional skin, non‐lesional skin and healthy skin were determined by qRT‐PCR assay. qRT‐PCR, real‐time quantitative fluorescence polymerase chain reaction; *, comparison between the two groups, *P* < 0.05; **, comparison between the two groups, *P* < 0.01.

### Expression of TLR4 in psoriasis

The expressions of TLR4 in psoriatic lesional skin, non‐lesional skin and healthy skin were detected by immunohistochemistry. It was shown that the expression of TLR4 was substantially high in psoriatic lesional skin. The TLR4‐positive cell rate and the number of positive cells per square millimetre in psoriatic lesional skin and non‐lesional skin were significantly higher than that in health skin (all *P* < 0.05) (Figs 2, 3). Moreover, the comparisons of the TLR4‐positive cell rate and the number of positive cells per square millimetre between psoriatic lesional skin and non‐lesional skin also showed statistical significance (all *P* < 0.05).

**Figure 2:** The expressions of TLR4 in psoriatic lesional skin, non‐lesional skin and healthy skin were detected by immunohistochemistry.

**Figure 3:** The TLR4‐positive cell rate and the number of positive cells per square millimetre in psoriatic lesional skin, non‐lesional skin and healthy skin. **(A)** the TLR4‐positive cell rate in psoriatic lesional skin, non‐lesional skin and healthy skin; **(B)** the number of positive cells per square millimetre in psoriatic lesional skin, non‐lesional skin and healthy skin. *, compared with healthy skin, *P* < 0.05; ^#^, compared with non‐lesional skin, *P* < 0.05.

### miR‐181b targeting TLR4

Prediction of miR‐181b targeting TLR4 was accomplished by the online software (http://www.targetscan.org). As can be seen in Figure 4A, miR‐181b had been presumed to interact with the 3′ untranslated region (3′UTR) of TLR4 based on software predictions. To demonstrate miR‐181b's function in targeting TLR4, the mutation (pMIR‐Report/TLR4‐mut 3′UTR) and wild‐type (pMIR‐Report/TLR4‐wt 3′UTR) sequences of the miR‐181b‐binding site of TLR4, with 3′UTR deleted, were inserted into reporter plasmids. Based on the dual‐luciferase reporter assay, Figure 4B has shown relative luciferase activity of HEKs cotransfected by miR‐181b mimics and wild‐type (TLR4‐wt) or mutation (TLR4‐mut) recombinant plasmids. It had been found that miR‐181b mimics had on obvious effect on the intensity of luciferase activity in mutation TLR4 (TLR4‐mut) plasmid group while the intensity of luciferase activity in wild‐type TLR4 (TLR4‐wt) plasmid group decreased by 45.9% with significant difference (*P* < 0.05), which indicates TLR4 is a direct target gene of miR‐181b in HEKs.

**Figure 4:** Verification of the relationship between miR‐181b and TLR4 by dual‐luciferase reporter assay. The luciferase expression at 48 h after transfection in HEKs, using TLR4‐3′UTR‐wt + miR‐181b mimic/negative control and TLR4‐3′UTR‐mut + miR‐181b mimic/negative control plasmids; HEKs, human epidermal keratinocytes; *, compared with negative control, *P* < 0.05.

### Regulation of miR‐181b on keratinocyte proliferation

In order to study effects of miR‐181b on the proliferation of HEKs, miR‐181b mimics or miR‐181b inhibitors were delivered into HEKs through liposomes. After transfection, the expressions of miR‐181b and TLR4 in HEKs were determined by qRT‐PCR assay and Western blotting respectively. Mitosis was examined using Brdu staining as markers and the number of marked cells was counted. As shown in Figure 5, the transfection of miR‐181b mimics led to an increase of miR‐181b expression but a decrease of TLR4 expression. Meanwhile, the expression of miR‐181b decreased, whereas that of TLR4 increased after HEKs transfected with miR‐181b inhibitors. The HEKs in all groups have been cultured for 3, 4 and 7 days correspondingly, the mitosis indexes and Brdu labelling indexes in the miR‐181b mimic group was remarkably decreased. However, in the miR‐181b inhibitor group, the mitosis indexes and Brdu labelling indexes significantly increased in comparison with other groups, while in HEKs transfected with miR‐181b inhibitor and siTLR4, the mitosis indexes and Brdu labelling indexes were significantly reduced, indicating that miR‐181b could target TLR4 to facilitate the proliferation of HEKs.

**Figure 5:** The expressions of miR‐181b and TLR4, mitosis, and the changes of the number of HEKs. (A) miR‐181b expression in each group; (B) TLR4 protein expression by western blotting; (C) quantitative histogram of TLR4 protein expression; (D) mitosis in each group; (E) the number of HEKs in each group; HEKs, human epidermal keratinocytes; LZRs, empty vectors; *, compared with the LZRs group, blank group and miR‐181b inhibitor + siTLR4 group, *P* < 0.05.

## Discussion

Psoriasis is an inflammatory and proliferous skin disease with a genetic predisposition and immune dysfunction tends to happen at keratinocytes which often show rapid cell proliferation, delayed differentiation and apoptosis 6. TLR4 has been shown to recognize lipopolysaccharides (LPS) of Gram‐negative bacteria, contributes to the defence to microbes on the skin surface and might be involved in the occurrence and development of psoriasis 33. Thus, this study, based on the prospective of genetics, first adopted the miR targeting technology to study the relationships among miR‐181b, TLR4 and HEKs in psoriasis.

By determination of expressions of miR‐181b and TLR4 in healthy skin, psoriatic non‐lesional skin and lesional skin, it has been found that the expressions of TLR4 in HEKs rise substantially with increased intensity of psoriatic lesion, which might be related to infection of skin lesions in patients with psoriasis. Several microorganisms (bacteria, fungi, etc.) have been implicated as triggers capable of initiating or exacerbating psoriasis 39, 40, 41, 42, among which LPS and peptidoglycan of Gram‐negative bacteria could be ligands of TLR4 on HEKs and further up‐regulate the TLR4 expression 33. In addition, the notable increase and decrease in TLR4 and miR‐181b expression correspondingly indicate miR‐181b's potential role in targeting TLR4 and intervening the proliferation and differentiation of HEKs in psoriatic lesion skin. According to relevant studies, miR‐181a has been proven to regulate expression of inflammatory mediators and factors by the TLR4 pathway 43, 44.

This study employed the dual‐luciferase reporter assay to verify that miR‐181b targets TLR4, probably undergoing similar mechanisms in miR‐181, by interacting with the 3′UTR of TLR4 mRNA to reduce TLR4 expression. Besides, it has also been shown that the expression of TLR4, mitotic index and Brdu labelling index markedly increased in HEKs transfected with miR‐181b inhibitors while those indexes were significantly decreased once cells were transfected with both miR‐181b mimics and siTLR4, illustrating the negative regulation of miR‐181b to TLR4 promoted the proliferation of HEKs. A potential mechanism has been proposed that high expression of TLR4 caused by low expression of miR‐181b results in excessive TLR4 which bind to LPS, interact with transforming growth factor β‐activated kinase 1 (TAK1) and activate nuclear factor‐κB (NF‐κB) 45. Upon generation of various effectors and cascade effects, many inflammatory mediators and cytokines, secreted by HEKs, stimulate the proliferation of HEKs in the occurrence and development of psoriasis 46, 47.

In conclusion, our study supported that miR‐181b can negatively regulate the proliferation of HEKs in psoriasis by targeting TLR4. With an increasing interest in ligands of TLR for psoriasis treatment, TLR agonists and antagonists (e.g. TLR7/9 antagonists) 48 revealed their wide applications in some immune‐mediated skin diseases including psoriasis. Hence, miR‐181b could provide new insights for seeking novel targets of treatment and prognosis of psoriasis. However, this study is limited because of certain limitations: (i) Role of miR‐181 and TLR4 in keratinocyte proliferation of psoriatic skin lesions and inflammation cannot be confirmed because of lack of determination of relevant inflammatory cytokines. (ii) Although the overexpression of miR‐181 is supposed to down‐regulate the expression of TLR4 and avoid excessive proliferation of HEKs, the model of miR‐181 overexpression has not yet been established. Further studies would be needed for validation of our results.

## Conflict of interest

None declared.
